The article "Application Effect of Dexmedetomidine and Dezocine in Patients Undergoing Lung Cancer Surgery under General Anesthesia and Analysis of Their Roles in Recovery Time and Cognitive Function" was published in 2022. Journal: Comput Math Methods Med.

# Application Effect of Dexmedetomidine and Dezocine in Patients Undergoing Lung Cancer Surgery under General Anesthesia and Analysis of Their Roles in Recovery Time and Cognitive Function

**DOI:** 10.1155/2022/9889534

**Published:** 2022-06-30

**Authors:** Jie Ding, Mengqi Zhu, Hu Lv, Jun Zhang, Wei Chen

**Affiliations:** ^1^Department of Anesthesiology, Fudan University Shanghai Cancer Center, Shanghai 200032, China; ^2^Department of Oncology, Shanghai Medical College, Fudan University, Shanghai 200032, China

## Abstract

**Objective:**

To explore the application influence of dexmedetomidine (DEX) and dezocine in patients undergoing lung cancer surgery under general anesthesia and analysis of their roles in recovery time and cognitive function.

**Methods:**

A total of 120 patients who accepted thoracoscopic pulmonary wedge resection in our hospital from November 2021 to April 2022 were selected and randomly divided into group A (*n* =60) and group B (*n* =60). DEX combined with dezocine-assisted anesthesia was performed to group A, and the equal dose of normal saline was administered to group B, so as to compare their inflammatory influence level, brain function, arterial blood gas index, and cognitive function.

**Results:**

Compared with group B, group A obtained significantly lower intraoperative and postoperative inflammatory factor levels (*P* < 0.001), better postoperative brain function and arterial blood gas index (*P* < 0.001), and lower Loewenstein Occupational Therapy Cognitive Assessment (LOTCA) scores after surgery (*P* < 0.001). Combining DEX with dezocine-assisted general anesthesia can improve the inflammatory factors level of patients undergoing lung cancer surgery and maintain their brain function and oxygen saturation, so that they have better postoperative cognitive function. Therefore, such anesthesia modality should be promoted in practice.

## 1. Introduction

Lung cancer is one of the most lethal malignancies, and in current practice, the prognosis of early-stage patients is improved mostly by thoracoscopic pulmonary wedge resection. However, surgical treatment involves general anesthesia, which can easily lead to immune response, stress reaction, and significant modification in hemodynamics during surgery, and in severe cases, hypoxaemia may even occur, causing injury in multiple organs such as the lung and brain and threatening patients' prognosis [1–3]. Administrating safe and effective adjuvant anesthetic drugs is an important measure to reduce intraoperative stress in patients, but studies have shown that drugs such as fentanyl can cause neuronal apoptosis in encephalic region [4], while isoflurane, etc. may affect the cognitive function [5], resulting in perioperative delirium; hence, with such limited function of the said drugs, the cardiocerebral vascular system of patients cannot be adequately protected. Dexmedetomidine (DEX) is a recent research hotspot in anesthesia, because it can not only alleviate vasoconstriction and blood pressure fluctuation induced by *α*1 epinephrine and improve the oxygen saturation for patients undergoing one-lung ventilation [6, 7], but also suppress the secretion frequency of noradrenaline by virtue of its high *α*2 epinephrine affinity, impair the stress response, and then protect the cardiocerebral vascular system in patients [8, 9]. On the basis of DEX, additionally administrating dezocine, a mixed opiate receptor agonist-antagonist, can have the effect of postoperative analgesia and lower the possibility of cognitive dysfunction.

The article "Application Effect of Dexmedetomidine and Dezocine in Patients Undergoing Lung Cancer Surgery under General Anesthesia and Analysis of Their Roles in Recovery Time and Cognitive Function" was published in 2022. Journal: Comput Math Methods Med.

There have been previous studies combining DEX with dezocine, but most attentive on their analgesic and sedative functions [10, 11], and none has explored their protective effects in assisting anesthesia on organ function in lung cancer patients who accepted surgery. Based on this, the actual application consequence was investigated in this study, with the results reported below.

The occurrence of cognitive dysfunction is related to many influences, and analysis of the mechanism of DEX combined with dezocine on cognitive dysfunction revealed that such combination can decrease the inflammatory response, protect multiple organs and systems, and greatly improve the brain function, lung function, cardiovascular system, and CNS.

## 2. Materials and Methods

### 2.1. General Information

120 patients who recognized thoracoscopic pulmonary wedge resection in our hospital from November 2021 to April 2022 were nominated and equally divided into group A and group B by random number way. No statistical differences were presented in the comparison of their general information (*P* > 0.05), see Table 1. The study was approved by the ethics committee of Fudan University Shanghai Cancer Center (approval No. 2111246-14; clinical trial registration No. ChiCTR2200056217).

### 2.2. Inclusion Criteria

The inclusion criteria of the study were as follows.

1. The patients, who had lung cancer and underwent endoscopy, signed the informed consent
2. The patients were at least 50 years old
3. The patients' physical status was class I-II according to the American Society of Anaesthesiologists (ASA) classification [12]
4. The patients' heart function was class I-II according to the New York Heart Association (NYHA) Functional Classification [10] and
5. The patients' Child-Pugh scores were class A and B [13]

### 2.3. Exclusion Criteria

The exclusion criteria for the patients of the study were as follows.

1. Age<50 years
2. BMI<18.5 or >40 kg/m^2^ [14]
3. Preoperative disturbance of consciousness and cognitive dysfunction
4. Coronary heart disease, severe arrhythmia, cardiorespiratory dysfunction, and cerebrovascular accidents
5. Anemia
6. Hyperglycemia
7. Liver and kidney dysfunction
8. Asthma, COPD, or presence of above moderate ventilatory dysfunction according to the lung function test results and
9. Speech disorder, seeing-hearing dysfunction

The article "Application Effect of Dexmedetomidine and Dezocine in Patients Undergoing Lung Cancer Surgery under General Anesthesia and Analysis of Their Roles in Recovery Time and Cognitive Function" was published in 2022. Journal: Comput Math Methods Med.

### 2.4. Methods

After entering the operating room, all patients were noticed for mean arterial pressure (MAP), heart rate (HR), electrocardiogram (ECG), and oxygen saturation, their vein passages were established, and a face mask was put on for oxygen inhalation. For patients in group A before surgery, 0.1 mg/kg of dezocine (manufacturer: Yangtze River Pharmaceutical (Group) Co., Ltd.; NMPA Approval No. H20080329) was diluted to 6 ml with normal saline and infused within 3 minutes, then the loading dose of 0.7 *μ*g/kg of DEX (manufacturer: Cisen Pharmaceutical Co., Ltd.; NMPA Approval No. H20130027) was diluted to 20 ml with normal saline and infused intravenously for 10 minutes. After the beginning of surgery, 0.3 *μ*g/(kg•h) of DEX was pump-injected at a constant rate to patients in group A, and at the same time, equal volume of normal saline was administered to patients in group B. For anesthesia induction of patients in the two groups, 0.03 mg/kg of midazolam (manufacturer: Jiangsu Nhwa Pharmaceutical Co., Ltd.; NMPA Approval No. H10980026), 0.3 *μ*g/kg of sufentanil (manufacturer: Yichang Humanwell Pharmaceutical Co., Ltd.; NMPA Approval No. H20054171), TCI 3~4 *μ*g/ml of propofol (manufacturer: Jiangsu Nhwa Pharmaceutical Co., Ltd.; NMPA Approval No. H20123138), and 0.6 mg/kg of rocuronium (manufacturer; Zhejiang Xianju Pharmaceutical Co., Ltd.; NMPA Approval No. H20123188) were administered. And for intraoperative anesthesia maintenance, 2.5-4 *μ*g/ml of propofol and TCI 2-4 ng/ml of remifentanil were administered, and additional 0.2 mg/kg of rocuronium could be given as needed.

Intraoperative parameters: tidal volume was 6 ml/kg, PEEP was 3-5 mmHg, air/oxygen mixture was given, oxygen flow rate was 2 L/min, EtCO_2_ was maintained at 35~45 mmHg, and Narcotrend was 40~60.

### 2.5. Observation Criteria

1. **Inflammatory factor level.** Before surgery (T_1_), during surgery (T_2_), at the end of surgery (T_3_), and 1 d after surgery (T_4_), 20 ml of vein blood was strained from the patients to extent the levels of interleukin-1*β* (IL-1*β*), interleukin-6 (IL-6), interleukin-10 (IL-10), and tumor necrosis factor-*α* (TNF-*α*) with the ELISA method (kits manufactured: Beijing Kewei Clinical Diagnostic Reagent Inc.; NMPA Approval No. S20060028)
2. **Brain function.** At T_1_, T_3_, and T_4_, 15 ml of vein blood was drawn from the patients to measure the levels of serum S100*β* protein and neuron-specific enolase (NSE) with the ELISA method, and their cerebral extraction of oxygen (CEO_2_) at the same moments was detected with the blood gas analyzer (GEM3000, Beckman Coulter Life Science, IN, USA; NMPA (I) 20082401894)
3. **Arterial blood gas indexes.** At T_1_, T_3_, and T_4_, the oxygen partial pressure (PaO_2_), carbon dioxide partial pressure (PaCO_2_), and lactate level (LAC) in patients were measured
4. **Cognitive function.** The cognitive function in patients at T_1_ and T_4_ was evaluated and compared with the Loewenstein Occupational Therapy Cognitive Assessment (LOTCA) [15, 16], which covered orientation (1-8 points), awareness (1-4 points), visuomotor construction (1-4 points), and thinking operations (1-4 points) and contained 20 items. The lower scores denoted that the patients' cognitive function was better

The article "Application Effect of Dexmedetomidine and Dezocine in Patients Undergoing Lung Cancer Surgery under General Anesthesia and Analysis of Their Roles in Recovery Time and Cognitive Function" was published in 2022. Journal: Comput Math Methods Med.

### 2.6. Statistical Processing

In this study, the data processing software was SPSS20.0, the picture drawing software was GraphPad Prism 7 (GraphPad Software, San Diego, USA), items included were enumeration data and measurement data, methods used were *X*^2^ test and *t*-test, and differences were considered statistically significant at *P* < 0.05.

## 3. Results

### 3.1. Comparison of Inflammatory Factor Levels

Group A obtained expressively lower intraoperative and postoperative inflammatory factor levels than group B (*P* < 0.001), see Figure 1.

Figure 1(a) shows the serum IL-1*β* level. At T_1_, the IL-1*β* levels of both groups were not significantly different (6.01 ± 0.98 vs 6.00 ± 0.89, *P* > 0.05); at T_2_, T_3_, and T_4_, the IL-1*β* levels of group A were remarkably lower than those of group B (9.54 ± 1.10 vs 14.65 ± 1.26, 6.98 ± 0.87 vs 9.10 ± 0.95, 6.75 ± 0.68 vs 8.65 ± 0.99, *P* < 0.001).

Figure 1(b) shows the serum IL-6 level. At T_1_, the IL-6 levels of both groups were not significantly different (59.65 ± 6.87 vs 59.21 ± 5.88, *P* > 0.05); at T_2_, T_3_, and T_4_, the IL-6 levels of group A were remarkably lower than those of group B (120.65 ± 12.98 vs 160.98 ± 15.98, 105.69 ± 8.65 vs 145.68 ± 12.68, 89.98 ± 5.87 vs 139.98 ± 10.65, *P* < 0.001).

Figure 1(c) shows the serum IL-10 level. At T_1_, the IL-10 levels of both groups were not significantly different (29.98 ± 2.15 vs 29.32 ± 2.44, *P* > 0.05); at T_2_, T_3_, and T_4_, the IL-10 levels of group A were remarkably lower than those of group B (50.68 ± 3.68 vs 62.98 ± 4.56, 37.21 ± 3.58 vs 45.68 ± 5.98, 34.21 ± 2.65 vs 41.65 ± 3.58, *P* < 0.001).

The article "Application Effect of Dexmedetomidine and Dezocine in Patients Undergoing Lung Cancer Surgery under General Anesthesia and Analysis of Their Roles in Recovery Time and Cognitive Function" was published in 2022. Journal: Comput Math Methods Med.

Figure 1(d) shows the serum TNF-*α* level. At T_1_, the TNF-*α* levels of both groups were not significantly different (12.54 ± 1.26 vs 12.65 ± 1.22, *P* > 0.05); at T_2_, T_3_, and T_4_, the TNF-*α* levels of group A were remarkably lower than those of group B (30.65 ± 3.68 vs 49.65 ± 4.98, 20.21 ± 1.68 vs 27.98 ± 2.10, 16.98 ± 1.11 vs 22.68 ± 1.24, *P* < 0.001).

### 3.2. Comparison of Brain Function

After surgery, the brain function of group A was clearly better than that of group B (*P* < 0.001), see Figure 2.

Figure 2(a) shows the serum S100*β* level. At T_1_, the S100*β* levels of both groups were not significantly different (0.49 ± 0.10 vs 0.48 ± 0.09, *P* > 0.05); at T_3_ and T_4_, the S100*β* levels of group A were remarkably lower than those of group B (1.10 ± 0.11 vs 1.89 ± 0.21, 0.76 ± 0.05 vs 1.54 ± 0.20, *P* < 0.001).

Figure 2(b) shows the serum NSE level. At T_1_, the NSE levels of both groups were not significantly different (5.12 ± 0.32 vs 5.11 ± 0.28, *P* > 0.05); at T_3_ and T_4_, the NSE levels of group A were remarkably lower than those of group B (12.98 ± 2.54 vs 19.65 ± 2.58, 15.11 ± 3.58 vs 18.26 ± 4.21, *P* < 0.001).

Figure 2(c) shows the CEO_2_ level. At T_1_, the CEO_2_ levels of both groups were not significantly different (36.54 ± 5.65 vs 36.98 ± 5.26, *P* > 0.05); at T_3_ and T_4_, the CEO_2_ levels of group A were remarkably lower than those of group B (38.21 ± 5.14 vs 49.65 ± 5.32, 41.98 ± 4.68 vs 48.99 ± 4.41, *P* < 0.001).

### 3.3. Comparison of Arterial Blood Gas Indexes

The postoperative arterial blood gas indexes of group A were significantly better than those of group B (*P* < 0.001), see Figure 3.

Figure 3(a) shows the PaO_2_ level. At T_1_, the PaO_2_ levels of both groups were not significantly different (100.56 ± 10.65 vs 101.98 ± 11.26, *P* > 0.05); at T_3_ and T_4_, the PaO_2_ levels of group A were remarkably higher than those of group B (380.65 ± 20.68 vs 328.98 ± 26.68, 100.23 ± 11.24 vs 82.65 ± 10.68, *P* < 0.001).

Figure 3(b) shows the PaCO_2_ level. At T_1_, the PaCO_2_ levels of both groups were not significantly different (43.65 ± 3.68 vs 43.96 ± 3.55, *P* > 0.05); at T_3_ and T_4_, the PaCO_2_ levels of group A were remarkably higher than those of group B (39.24 ± 3.21 vs 30.68 ± 2.88, 42.10 ± 2.65 vs 36.98 ± 3.54, *P* < 0.001).

Figure 3(c) shows the LAC level. At T_1_, the LAC levels of both groups were not significantly different (0.87 ± 0.10 vs 0.89 ± 0.09, *P* > 0.05); at T_3_ and T_4_, the LAC levels of group A were remarkably lower than those of group B (1.32 ± 0.11 vs 1.42 ± 0.10, 0.99 ± 0.10 vs 1.20 ± 0.15, *P* < 0.001).

The article "Application Effect of Dexmedetomidine and Dezocine in Patients Undergoing Lung Cancer Surgery under General Anesthesia and Analysis of Their Roles in Recovery Time and Cognitive Function" was published in 2022. Journal: Comput Math Methods Med.

### 3.4. Comparison of Cognitive Function

After surgery, group A obtained significantly lower LOTCA score than group B (*P* < 0.001), see Table 2.

## 4. Discussion

Surgery can efficiently resect tumor tissue and dissect metastatic lymph nodes in lung cancer patients, but it is moderately traumatic and can trigger nonspecific reactions in the body, resulting in hemodynamics changes and fluctuating vital signs in patients, and even convincing ischemic damage in severe cases, which in turn elevates the inflammatory level and makes patients experience multiple complications such as organ dysfunction. Cognitive dysfunction is one of the most common postoperative complications of lung cancer [17], which increases the late mortality of patients. Factors such as stress reaction, surgical trauma, deterioration of cerebrovascular microcirculation, and hypoxemia can raise the possibility of cognitive dysfunction [18]. Anesthetic drugs can directly affect this complication by acting on the central nervous system (CNS) [19], so selecting suitable anesthetic adjuncts is beneficial to reduce the odds of cognitive dysfunction and improve patient outcomes.

The anesthetic drugs selected in this study were DEX, a widely used sedative agent in the clinic with significant efficacy in sedation, analgesia, and reducing stress reactions, and dezocine, a strong analgesic [20]. The study results showed that after surgery, group A obtained lower scores on LOTCA (with additional items such as spatial perception and thinking operations compared with the mini-mental state examination (MMSE)) than group B (*P* < 0.001), fully demonstrating that the cognitive function of group A was more ideal. Based on the results, it could be estimated that the mechanisms of lowering the odds of cognitive function by combining DEX with dezocine were as follows.

1. DEX, an *α*_2_-adrenoceptor agonist, could suppress the sympathetic nerve impulse in CNS and lift the activity of vagus nerve, thereby lowering the odds of hypotension while maintaining the cerebral oxygen metabolism, alleviating cerebral perfusion damage, and then protecting the brain function. The S100*β* (a nerve cell injury marker) and NSE (a soluble plasmosin) selected in this study could enter the peripheral blood when the nerve cells were injured. The results presented that the postoperative brain function indexes of group A were significantly better than those of group B (*P* < 0.001), denoting that DEX well-protected the brain function
2. When activating the *α*_2_ adrenergic receptor agonist, DEX could lower the secretion frequency of noradrenaline and control the autonomic nervous reflex, while dezocine, the opiate receptor agonist-antagonist, could maintain stable hemodynamics, so combining the two could sufficiently alleviate the perioperative stress response of lung cancer patients and lower their angiotensin II level [21]
3. Surgical stress caused the release of TNF-*α* and other inflammatory factors and inflammatory reactions could damage the cardiocerebral vascular system in patients and trigger astrocyte activation in the CNS. Moon T and other scholars found that TNF-*α* could worsen cognitive function in patients [22], while the study by scholars Gao S et al. showed that DEX reduced the release of inflammatory mediators in toxin-induced shock rats [23], decreased the level of TNF-*α* and other inflammatory factors, and avoided mediating the memory loss reactions in CNS. This study also presented that group A obtained significantly lower intraoperative and postoperative inflammatory factor levels than group B (*P* < 0.001), which was consistent with the general findings in academia
4. Lung cancer surgery required one-lung ventilation with endotracheal intubation, which impaired the patients' intra-pulmonary gas diffusion function and reduced the gas exchange capacity between pulmonary alveolar and pulmonary capillary, so the patients were prone to hypoxaemia triggered by oxygenation decline. Scholar S. L. Zong research found that DEX, which had a slight effect on the respiratory center, was able to improve the arterial blood gas indicators and alleviate pulmonary infection in patients [24], and the respiration would not be inhibited by low-dose dezocine, so the combination of the two drugs could effectively maintain respiratory movement, alleviate lung injury, and improve lung and brain microcirculation with better CeO_2_; accordingly, the rate of cognitive impairment was reduced

The occurrence of cognitive dysfunction is related to many factors, and analysis of the mechanism of DEX combined with dezocine on cognitive dysfunction revealed that such combination can reduce the inflammatory response, protect multiple organs and systems, and greatly improve the brain function, lung function, cardiovascular system, and CNS. At present, most Chinese lung cancer patients are elderly who have poor body organs combined with multiple complications and are extremely prone to postoperative cognitive dysfunction and organ dysfunction. With DEX and dezocine-assisted anesthesia, the odds of postoperative complications can be efficiently reduced and the long-term prognosis of patients can be guaranteed. It should be noted that no adverse consequence-related research was done in this study, and general findings in academia showed that the combination did not increase the chance of adverse effects, but whether the applied dose of DEX and dezocine could affect the safety needs to be further explored.

The article "Application Effect of Dexmedetomidine and Dezocine in Patients Undergoing Lung Cancer Surgery under General Anesthesia and Analysis of Their Roles in Recovery Time and Cognitive Function" was published in 2022. Journal: Comput Math Methods Med.

## 5. Conclusion

Combining DEX with dezocine-assisted anesthesia can lower the perioperative inflammatory factor level, guarantee the brain function and oxygen saturation, and ensure better postoperative cognitive function in lung cancer patients undergoing surgery, which should be promoted in practice.

## Figures and Tables

**Figure 1:** Comparison of inflammatory factor levels ($\bar{x}\pm s$). Note: In Figure 1, the horizontal axis from left to right showed T_1_, T_2_, T_3_, and T_4_, the lines with dots denoted group A, and the lines with blocks denoted group B.

**Figure 2:** Comparison of brain function ($\bar{x}\pm s$). Note: In Figure 2, the horizontal axis showed T_1_, T_3_, and T_4_, the black areas denoted group A, and the gray areas denoted group B.

**Figure 3:** Comparison of arterial blood gas indexes ($\bar{x}\pm s$). Note: In Figure 3, the horizontal axis from left to right indicated T_1_, T_3_, and T_4_, the lines with dots denoted group A, and the lines with blocks denoted group B.

**Table 1:** Comparison of patients' general information.

Group	Group A (*n* =60)	Group B (*n* =60)	*X* ^2^/*t*	*P*
Gender			0.03	0.85
Male	35	36		
Female	25	24		
Age (years old)				
Range	60-76	60-74		
Mean age	68.26 ± 5.54	68.52 ± 5.21	0.26	0.79
Mean body weight (kg)	54.98 ± 2.65	54.54 ± 2.57	0.92	0.36
Complications				
Chronic bronchitis	8	9	0.07	0.79
Chronic obstructive pulmonary disease	10	9	0.06	0.80
Mean duration of disease (years)	4.21 ± 0.68	4.10 ± 0.56	0.97	0.33
Anesthesia grade			0.04	0.85
I	38	39		
II	22	21		
Tumor stage				
II	21	22	0.04	0.85
III	25	24	0.03	0.85
IV	14	14	0.00	1.00
Mean BMI (kg/m^2^)	22.65 ± 2.51	22.68 ± 2.50	0.07	0.95
Place of residence			0.04	0.85
Urban area	40	41		
Rural area	20	19		
Monthly income (yuan)			0.04	0.85
≥4,000	38	37		
<4,000	22	23		
Living habit				
Smoking history	42	40	0.15	0.69
Drinking history	35	34	0.03	0.85
Educational degree			0.14	0.71
Senior high school and below	23	25		
College and above	37	35		

**Table 2:** Comparison of LOTCA scores ($\bar{\text{x}}\pm s$, points).

Category	Group A		Group B		*t*	*P*
LOTCA	T_1_	79.65 ± 5.98	T_1_	79.54 ± 5.24	0.11	0.92
	T_4_	48.65 ± 5.62	T_4_	60.11 ± 5.36	11.43	< 0.001
	*t*	29.261	*t*	20.078		
	*P*	< 0.001	*P*	< 0.001		

## Data Availability

Data to support the findings of this study is available on reasonable request from the corresponding author.
